# Anti-GBM of Pregnancy: Acute Renal Failure Resolved after Spontaneous Abortion, Plasma Exchange, Hemodialysis, and Steroids

**DOI:** 10.1155/2014/243746

**Published:** 2014-06-24

**Authors:** Mohammed Muqeet Adnan, Jordan Morton, Syed Hashmi, Sufyan Abdul Mujeeb, William Kern, Benjamin Jr. Cowley

**Affiliations:** ^1^Department of Internal Medicine, University of Oklahoma Health Sciences Center, Oklahoma City, OK 73117, USA; ^2^University of Illinois at Chicago, Chicago, IL 60612, USA; ^3^Department of Pathology, University of Oklahoma Health Sciences Center, Oklahoma City, OK 73117, USA; ^4^Department of Nephrology, University of Oklahoma Health Sciences Center, Oklahoma City, OK 73117, USA

## Abstract

Antiglomerular basement membrane disease presenting during pregnancy is very uncommon. We present a case of a pregnant female who presented with acute renal failure needing dialysis from Goodpasture's disease. She responded very well to just plasma exchange, high dose steroids, and hemodialysis. Cyclophosphamide was never started on this patient. She had a spontaneous abortion in her 8th week of pregnancy and henceforth did very well to regain her renal function. Patient became hemodialysis independent at 2 months and returned to her baseline kidney function at 6 months. We present this remarkable case of recovery from acute renal failure in a patient with anti-GBM disease. We think the flare-up of renal failure was pregnancy related which resolved after spontaneous abortion.

## 1. Case

A 17-year-old 6-week-pregnant female was admitted for nausea and vomiting for a suspected morning sickness. At admission patient was found to have a mild fever of 99 F, hemoglobin of 6.5 mg/dL, and serum creatinine at 6.47 mg/dL. Baseline creatinine six months earlier was 0.6 mg/dL. A thrombotic thrombocytopenic purpura was suspected despite normal platelets and hence she was admitted to the hospital for further workup. Vital signs at admission were temperature of 99 F, heart rate of 90–100 beats per minute, respiratory rate of 14 cycles per minute, and blood pressure of 120–130/80 s. Physical exam was consistent with a normal female who was moderately built without any evidence of fluid overload like raised jugular venous distension and facial or leg edema. Heart and lung exam were within normal limits. Patient's neurological exam was intact. Laboratory findings were as follows: hemoglobin 6.51 mg/dL, white blood cell count  10.3 k/mm^3^, platelets 384 k/mm^3^, sodium 136 mEq/L, potassium 4.4 mEq/L, chloride 107 mEq/L, bicarbonate 21 mEq/L, blood urea nitrogen 26 mg/dL, and creatinine 6.47 mg/dL. Iron studies showed iron deficiency anemia with iron of 25 mcg/dL, total iron binding capacity of 185 mcg/dL, iron saturation of 14%, and transferrin of 132 mg/dL. Urine analysis at admission showed urine pH of 6.5, specific gravity of 1.009, urine protein of 2+, and urine blood of 3+ with too numerous RBCs to count; urine glucose, ketones, bilirubin, and leukocyte esterase were all negative. Other tests that were ordered were antiglomerular basement membrane antibodies which were high at 156 units. Complement C3 and C4 levels were high at 195 and 57, respectively. Antineutrophil antibody, antineutrophil cytoplasmic antibody, antiproteinase 3, anti-Smith, and ds DNA were negative. Other miscellaneous lab tests like HIV antibody, hepatitis A IgM antibody, hepatitis B surface antigen, hepatitis B core IgM antibody, hepatitis C antibody, and antistreptolysin O Ab were all negative.

On the second day of hospitalization the patient underwent a kidney biopsy for a suspected anti-GBM disease. The preliminary biopsy results based on the hematoxylin and eosin stains showed acute necrotizing and crescentic glomerulonephritis. Final pathology results showed acute crescentic glomerulonephritis with no globally obsolescent glomeruli, moderate interstitial inflammation, and mild fibrosis. The final images of the pathology slides are shown in Figures 1 and 2.

Patient was given 2 units of PRBC after admission with a posttransfusion Hb at 8.9 mg/dL. Peripheral smear did not show any schistocytes and hence the diagnosis of TTP was ruled out. All the labs and pathology suggested acute anti-GBM disease. On hospital day 3 plasmapheresis and high dose methylprednisolone at 1 gm/day were begun. See Figure 3 for creatinine trend. Creatinine peaked to 7.48 on day 5 and the patient was slowly becoming oliguric, showing sign of fluid overload with pedal edema and lung crackles on physical exam and hence was initiated on intermittent hemodialysis on day 5 of hospitalization. Patient received a total of 3 doses of methylprednisolone at 1 gm/day and then was started on prednisone at 60 mg/day from day 4.

To prevent further renal injury the option of adding cyclophosphamide was discussed but was not done due to possible fetal adverse outcomes. On day 17 of hospitalization the patient had a spontaneous abortion. After abortion cyclophosphamide was not started due to patient's request and hence she was managed with plasmapheresis and high dose prednisone. The plasmapheresis sessions were started on day 3 and continued daily until discharge (day 25). Traditional plasmapheresis with albumin replacement and sometimes 70% albumin with 30% normal saline replacement that lasted for 3 hours every day was the technique used. She was never started on cyclophosphamide and slowly became hemodialysis independent in about 2 months from discharge. At about 6 months from discharge the patient lost to follow up. It was deemed that the acute anti-GBM flare-up was pregnancy related.

## 2. Discussion

Anti-GBM disease is an immune complex small vessel vasculitis [1]. The disease is characterized by immune complex deposition in places where there is basement membrane, that is, glomeruli or pulmonary capillaries. Patients develop autoantibodies to the basement membrane which are hence called anti-GBM antibodies; these antibodies when binding to the basement membrane activate the classical pathway of the complement system and hence then start a neutrophilic inflammation which results in a crescentic glomerulonephritis [1]. Anti-GBM disease generally produces a rapidly progressive glomerulonephritis which despite treatment with cytotoxic agents and steroids results in only one-third of patients surviving this rapidly fatal disease [1]. Anti-GBM of pregnancy is very uncommon. So far about 5 cases have been reported in the literature. Three cases were briefly described by Al Harbi et al. in their case report [2]. A fifth one was recently reported by Nair et al. [3].

*Cases Reported So Far*

1. Nilssen et al., in their report of 4 cases, describe a pregnant patient who developed acute renal failure postpartum and never recovered despite steroids, plasma exchange, and cyclophosphamide and was dialysis dependent [2, 4].
2. Yankowitz et al. describe a patient who had a diagnosis of Goodpasture's but with immunosuppressive therapy her anti-GBM levels became negative and the patient had a successful delivery [2, 5].
3. Deubner et al. describe a case of anti-GBM disease which was diagnosed postpartum and they attribute that the placenta might have been responsible in controlling the disease while the patient was pregnant [2, 6].
4. Al Harbi et al. described a 30-year-old female who needed dialysis during her pregnancy until delivery from RPGN due to anti-GBM disease [2].
5. Nair et al. describe a case of anti-GBM diagnosed during pregnancy which responded to plasma exchange and steroids; the pregnancy was terminated at 15 weeks and after termination the patient's renal failure returned to normal limits with plasma exchange and steroids [3].

We describe a pregnant female who was found to have acute renal failure during her 6th week of pregnancy. Based on the case reports, be it postpartum or antepartum, anti-GBM disease that generally presents during or after pregnancy is severe enough to cause oliguric renal failure. Treatment of anti-GBM causing rapidly progressing glomerulonephritis is generally plasma exchange, high dose steroids, and cytotoxic agents like cyclophosphamide. It is generally very unusual to have a renal recovery if kidney failure is so severe that requires frequent dialysis to maintain electrolyte equilibrium and euvolemia.

We treated our patient with plasma exchange and high dose steroids and because the renal failure was worsening we had to start hemodialysis. Despite all measures spontaneous abortion could not be prevented. The patient never wanted to use any cytotoxic drugs and hence they were never initiated. She received several plasma exchanges while being in the hospital for more than a month. The anti-GBM levels came down and were almost undetectable prior to discharge (Figure 4). The renal recovery was remarkable and as an outpatient the patient required less frequent hemodialysis, her steroids were completely tapered, and the kidney function was back to baseline. Pregnancy in general is a very high risk state and exacerbation of autoimmune diseases is a very common phenomenon that occurs during pregnancy. We think that our patient developed a rapidly progressive glomerulonephritis from being pregnant and once the trigger was removed, that is, spontaneous abortion, her kidney function started to return to normal along with the multiple treatment regimens which were washing out the antibodies to the glomerular basement membrane. This case is very unique with a remarkable recovery and we think people who have been diagnosed with anti-GBM of pregnancy need very close follow-up with repeated renal function tests and frequent glomerular filtration rate assessment. They will possibly need more immunosuppression prior to planning a pregnancy as an exacerbation can occur with another pregnancy [5].

## Figures and Tables

**Figure 1:** Immunofluorescence staining shows linear GBM staining for IgG consistent with Goodpasture's disease.

**Figure 2:** H&E stains showing crescentic glomerulonephritis with moderate interstitial inflammation and mild fibrosis with no evidence of vasculitis.

**Figure 3:** Graph showing trend of creatinine (mg/dL) while in the hospital. Plasmapheresis and corticosteroids were initiated on day 3. Hemodialysis was initiated on day 5. Daily plasmapheresis with high dose prednisone at 60 mg/day was continued until discharge. Hemodialysis was done intermittently three times a week.

**Figure 4:** Trend in the anti-GBM levels with plasmapheresis and high dose prednisone.
